The article "High Doses of Silica Nanoparticles Obtained by Microemulsion and Green Routes Compromise Human Alveolar Cells Morphology and Stiffness Differently" was published in 2022. Journal: Bioinorg Chem Appl.

# High Doses of Silica Nanoparticles Obtained by Microemulsion and Green Routes Compromise Human Alveolar Cells Morphology and Stiffness Differently

**DOI:** 10.1155/2022/2343167

**Published:** 2022-01-31

**Authors:** Valeria De Matteis, Mariafrancesca Cascione, Agnese De Luca, Daniela Erminia Manno, Rosaria Rinaldi

**Affiliations:** Department of Mathematics and Physics “Ennio De Giorgi”, University of Salento, Via Arnesano, Lecce 73100, Italy

## Abstract

Among all the inorganic nanomaterials used in commercial products, industry, and medicine, the amorphous silica nanoparticles (SiO_2_ NPs) appeared to be often tolerated in living organisms. However, despite several toxicity studies, some concerns about the exposure to high doses of SiO_2_ NPs with different sizes were raised. Then, we used the microemulsion method to obtain stable SiO_2_ NPs having different sizes (110 nm, 50 nm, and 25 nm). In addition, a new one-pot green synthetic route using leaves extract of *Laurus nobilis* was performed, obtaining monodispersed ultrasmall SiO_2_ NPs without the use of dangerous chemicals. The NPs achieved by microemulsion were further functionalized with amino groups making the NPs surface positively charged. Then, high doses of SiO_2_ NPs (1 mg/mL and 3 mg/mL) achieved from the two routes, having different sizes and surface charges, were used to assess their impact on human alveolar cells (A549), being the best cell model mimicking the inhalation route. Cell viability and caspase-3 induction were analyzed as well as the cellular uptake, obtaining that the smallest (25 nm) and positive-charged NPs were more able to induce cytotoxicity, reaching values of about 60% of cell death. Surprisingly, cells incubated with green SiO_2_ NPs did not show strong toxicity, and 70% of them remained vital. This result was unusual for ultrasmall nanoobjects, generally highly toxic. The actin reorganization, nuclear morphology alteration, and cell membrane elasticity analyses confirmed the trend achieved from the biological assays. The obtained data demonstrate that the increase in cellular softness, i.e., the decrease in Young's modulus, could be associated with the smaller and positive NPs, recording values of about 3 kPa. On the contrary, green NPs triggered a slight decrease of stiffness values (c.a. 6 kPa) compared to the untreated cells (c.a. 8 kPa). As the softer cells were implicated in cancer progression and metastasization, this evidence strongly supported the idea of a link between the cell elasticity and physicochemical properties of NPs that, in turn, influenced the interaction with the cell membrane. Thus, the green SiO_2_ NPs compromised cells to a lesser extent than the other SiO_2_ NPs types. In this scenario, the elasticity evaluation could be an interesting tool to understand the toxicity of NPs with the aim of predicting some pathological phenomena associated with their exposure.

The article "High Doses of Silica Nanoparticles Obtained by Microemulsion and Green Routes Compromise Human Alveolar Cells Morphology and Stiffness Differently" was published in 2022. Journal: Bioinorg Chem Appl.

## 1. Introduction

SiO_2_ NPs are considered the most popular nanomaterials thanks to their unique properties [1]; they are easy to obtain through different chemical approaches, the surface can be functionalized with several chemical groups [2], and the size can be customized [3]. These NPs are widely used in the field of nanomedicine [4, 5], cosmetics [6], food additives, and packaging [7], as well as in many household products, such as toothpaste and paints [8, 9]. In addition, they are present as components of particulate matter (PM) [10]. Although the major toxicity was found when living organisms were exposed to crystalline form of SiO_2_ [11], for the correspondent amorphous forms, conflicting data are available in the literature regarding their toxicity [12]. Generally, the microsize and low doses seem to be the two parameters that make SiO_2_ NPs biocompatible [13, 14], as the small size is associated with the larger surface area and then higher chemical reactivity [15]. Then, it is important to know the toxic behavior of the NPs smaller than 100 nm; these are able to enter into the cells by both passive diffusion and active endocytosis, reaching the different cellular compartments such as cytoplasm and organelles [16, 17]. In order to mimic the inhalation route, Gonzales et al. [18] exposed A549 to SiO_2_ NPs having 16 nm, 60 nm, and 104 nm of size. The viability study was performed using three NPs concentrations (the maximum value was 165.9 *μ*g/mL) for 24 h showing size-dependent cytotoxicity. The same results were obtained by another work in which the SiO_2_ NPs (6 nm) induced apoptosis activation contrary to the same having larger sizes, that is, 15 and 30 nm [19]. In addition, the adverse effects were dependent on the NPs concentration, which normally was tested as *μ*g/mL. Furthermore, the toxicity is also influenced by the surface functionalization that defines a specific surface charge; for example, the conjugation with amino-type groups makes the SiO_2_ NPs positive. Charged NPs (positive or negative) are more able to adsorb human serum proteins in a different manner with respect to neutral NPs. In particular, the negative charged NPs were more efficient in binding proteins compared to the positive counterpart [20]. Then, the protein corona formation and its thickness can be crucial elements for cell uptake efficiency. Additionally, Kokkinopoulou et al. [21] concluded that the negative NPs functionalized with carboxyl groups formed larger protein corona compared to the amine-decorated NPs. Once in the cell, the amorphous SiO_2_ NPs are able to trigger the Reactive Oxygen Species (ROS) generation: their overproduction is connected to oxidative stress, whereas the low ROS amount contributes to regulating some cellular functions, extending the cellular lifetime [22, 23]. Despite the fact that the potential toxicity of SiO_2_ NPs has been investigated in countless studies, only a few works have analyzed the cell behavior when they are exposed to high doses (in terms of milligrams) of SiO_2_ NPs. This assessment is necessary since these kinds of NPs are largely used in different fields of application, including nanomedicine. In addition, beyond the conventional biological assays, few studies have focused on the cellular mechanical response following NPs exposure [24]. Any alteration of cell elasticity, in terms of Young's modulus [25, 26], induces several consequences on the cellular functions [27]. Precisely, the softer cell membrane is associated with cell spreading and migration, whereas the stiffer membrane can inhibit some physiological phenomena like differentiation [28, 29].

The article "High Doses of Silica Nanoparticles Obtained by Microemulsion and Green Routes Compromise Human Alveolar Cells Morphology and Stiffness Differently" was published in 2022. Journal: Bioinorg Chem Appl.

Here, we assess the toxicity induced by high doses (1 mg/mL and 5 mg/mL) of SiO_2_ NPs on A549 cells after 24 h and 48 h of time exposure. Specifically, we used three sizes of SiO_2_ NPs (i.e., 110, 50, and 25 nm), both negative (bare) and positive charged (functionalized with amino groups), obtained by the microemulsion method. In addition, we compared cytotoxic data with the ones obtained after exposure to amorphous SiO_2_ NPs synthetized by green route using *Laurus nobilis* extract. The “green” route is based on the use of polyphenols contained in leaves, allowing for the production of NPs with high yield without the use of toxic chemicals, especially cyclohexane and ammonia. In addition, it permits us to reduce both the energy-associated cost of synthesis and the waste products [30].

We evaluated the viability, apoptosis induction, and uptake, as well as morphological alterations of the actin cytoskeleton and nuclei (strictly connected to the cell damage), analyzing the morphological parameters. In addition, a careful evaluation of cell membrane elasticity was performed to assess the potential impact of the different types of SiO_2_ NPs on Young's modulus values using Atomic Force Microscopy (AFM). Our results demonstrated a size and surface charge-dependent toxicity using NPs achieved by the microemulsion route. On the contrary, few adverse effects were unexpectedly measured when green NPs were applied, despite their ultrasmall size (c.a. 4 nm). These results add important knowledge in green methods development with the aim of obtaining nanomaterials with low toxicity for their safe use in nanomedicine.

The article "High Doses of Silica Nanoparticles Obtained by Microemulsion and Green Routes Compromise Human Alveolar Cells Morphology and Stiffness Differently" was published in 2022. Journal: Bioinorg Chem Appl.

## 2. Materials and Methods

### 2.1. Reagents

Triton X-100, cyclohexane (≥99.8%), tetraethyl orthosilicate (TEOS ≥99.0%), ammonium hydroxide (NH_4_OH, 28.0–30.0%), aminopropyltriethoxysilane (APTES), ethanol absolute (≥99.8%), nitric acid (HNO_3_ > 90%), hydrochloric acid (HCl 37%), Dulbecco's Modified Eagle's Medium-high glucose (DMEM), Leibovitz (L15) medium, fetal bovine serum (FBS), penicillin-streptomycin, dimethyl sulfoxide (DMSO), WST-8 assay, phosphate buffer saline (PBS), silicon standard, 4′,6-diamidine-2′-phenylindole dihydrochloride (DAPI), trypsin, glutaraldehyde, FITC-phalloidin, and caspase-3 colorimetric assay kit (CASP-3-C) were purchased from Sigma Aldrich, Dorset, UK. Petri dishes and multiwell were purchased from Corning® Costar®. All the reagents were used as received without further purification.

### 2.2. Synthesis of Silica NPs (110 nm, 50 nm, and 25 nm) by the Microemulsion Route

The synthetic procedure to obtain the three sizes of NPs was conducted using the method described in [31] with some modifications. The 25 nm SiO_2_ NPs was obtained by ternary microemulsion mixing 800 *μ*L of Triton X-100, 3.75 mL of cyclohexane, 170 *μ*L of water, 40 *μ*L of TEOS, and 70 *μ*L of NH_4_OH. Then, the solution was left under stirring for 24 h. After this time, the reaction was stopped using absolute ethanol. A centrifugation step (4000 rpm for 1 hour) was carried out to obtain SiO_2_ NPs in the pellet. After this step, NPs were washed five times using a mix of ethanol and water by means of a minicentrifuge at a speed of 13.000 rpm for 20 minutes/wash route. The syntheses of 50 nm and 110 nm of SiO_2_ NPs were conducted using the quaternary w/o microemulsion using pentanol for 50 nm NPs and butanol for 110 nm. Briefly, 800 *μ*L of Triton X-100, 3.75 mL of cyclohexane, and 800 *μ*L of alcohol were mixed and stirred with a vortex in order to obtain a clear solution. After mixing, 170 *μ*L of water, 40 *μ*L of TEOS, and 35 *μ*L of NH_4_OH were added. The following steps were the same described for the 25 nm SiO_2_ NPs. A general procedure for SiO_2_ NPs synthesis in microemulsion is schematized in Figure 1.

### 2.3. Functionalization of the SiO_2_ NPs Surface

SiO_2_ NPs were dispersed in a freshly prepared 5% (v/v) solution of APTES and absolute ethanol. Then the mix was stirred overnight. After reaction, NPs were collected by two centrifugation steps (13000 rpm, 20 min), washed 5 times with ethanol and water (1 : 1), and finally redispersed in MilliQ water. A schematic representation of the APTES functionalization route is represented in Figure 2.

The article "High Doses of Silica Nanoparticles Obtained by Microemulsion and Green Routes Compromise Human Alveolar Cells Morphology and Stiffness Differently" was published in 2022. Journal: Bioinorg Chem Appl.

### 2.4. Green Synthesis of SiO_2_ NPs

#### 2.4.1. Preparation of the Leaves Extract

The leaves of *Laurus nobilis* were harvested during the winter. Numerous washes with MilliQ water were made in order to eliminate any pollutants or other contaminants deposited on the leaves. After drying, leaves were cut, and 20 g of them was added to 200 mL of MilliQ water in a beaker placed on a hotplate until boiling. After this step, the mix was left to boil for 20 minutes. The extract was then cooled to room temperature in the dark and then filtered using Whatman filter paper.

#### 2.4.2. Synthetic Procedure

For the green synthesis, 2 mL of TEOS, 2 mL of ethanol-Triton-X solution (in a ratio of 1 : 0.1), and 2 mL of *Laurus nobilis* leaves extract were mixed and then left to stir for 24 h. The next day, the NPs were recovered by centrifugation (4500 rpm, 30 min, 25°C), and the surfactant and unreacted molecules were washed away from the resulting SiO_2_ NPs precipitate. Then, the NPs were washed 5–6 times with a solution of acetone and water (1 : 1) to purify the nanomaterials. A schematic representation of the one-pot synthetic procedure is reported in Figure 3.

### 2.5. Lyophilization of SiO_2_ NPs

The final suspensions of pure SiO_2_ NPs were frozen at −20°C for 3 h, and the resulting solids were freeze-dried using Alpha 1–2 LD plus (Christ Gefriertrocknungsanlagen GmbH, Germany) for 24 h to obtain SiO_2_ NPs white powder.

### 2.6. Characterization of SiO_2_ NPs

#### 2.6.1. Transmission Electron Microscopy (TEM) Analysis

TEM images and electron diffraction patterns were taken using a Hitachi 7700 transmission electron microscope operating at 120 kV. The solutions of SiO_2_ NPs achieved from the microemulsion approach and SiO_2_ NPs obtained by the green route were dropped onto 600-mesh copper grids coated with carbon film. After a slow drying in the air, the samples were ready for the observations at TEM.

#### 2.6.2. DLS and Zeta Potential in Water and in DMEM

The DLS and *ζ*-potential acquisitions were recorded by a Zetasizer Nano-ZS having a HeNe laser (4.0 mW) working at 633 nm detector (ZEN3600, Malvern Instruments Ltd., UK) in aqueous solutions (25°C, pH 7) and in DMEM. NPs size statistical distribution was measured on 70 NPs fitted by a normal Gaussian function using ImageJ software.

### 2.7. Cell Culture

A549 (ATCC® CCL-185™) were maintained in DMEM with 50 *μ*M glutamine, supplemented with 100 U/mL penicillin and 100 mg/mL streptomycin and 10% of FBS. Cells were incubated in a humidified controlled atmosphere with a 95 to 5% ratio of air/CO_2_, at 37°C.

### 2.8. Viability Assay

A549 cells were seeded in 96-well microplates at a concentration of 5 × 10^3^ cells/well. After 24 h of stabilization, SiO_2_ NPs 110 nm (−), SiO_2_ NPs 110 nm (+), SiO_2_ NPs 50 nm (−), SiO_2_ NPs 50 nm (+), SiO_2_ NPs 25 nm (−), SiO_2_ NPs 25 nm (+), and green SiO_2_ NPs stock solutions were added to the cell medium at 1 mg/mL and 5 mg/mL. Cells were incubated for 24 h and 48 h. At the endpoints, cell viability was measured using a standard WST-8 assay. Assays were performed following the procedure previously described in De Matteis et al. [17]. Data were expressed as mean ± SD.

The article "High Doses of Silica Nanoparticles Obtained by Microemulsion and Green Routes Compromise Human Alveolar Cells Morphology and Stiffness Differently" was published in 2022. Journal: Bioinorg Chem Appl.

### 2.9. Internalization of SiO_2_ NPs in a549 Cells

1 × 10^5^ of A549 cells were seeded in 1 mL of the DMEM in a 6-well plate. After 24 h of stabilization, the medium was replaced with a fresh medium containing SiO_2_ NPs 110 nm (−), SiO_2_ NPs 110 nm (+), SiO_2_ NPs 50 nm (−), SiO_2_ NPs 50 nm (+), SiO_2_ NPs 25 nm (−), SiO_2_ NPs 25 nm (+), and green SiO_2_ NPs at a concentration of 1 mg/mL and 5 mg/mL for 24 h and 48 h. Then, the culture medium was discarded, and cells were washed with PBS. An automatic cell counting chamber was used to count cells after trypsin treatment. 360.000 cells were suspended in 200 *μ*L of MilliQ water and digested by *aqua regia* (HNO_3_ : HCl, 1 : 3). The solution was diluted, and elemental analysis was carried out using an ICP-OES Perkin Elmer AVIO 500 to evaluate the Si content.

### 2.10. Caspase-3 Assay

The activity of caspase-3 was determined using a colorimetric assay kit. Briefly, A549 cells (5.000 cells/well) were incubated with SiO_2_ NPs 110 nm (−), SiO_2_ NPs 110 nm (+), SiO_2_ NPs 50 nm (−), SiO_2_ NPs 50 nm (+), SiO_2_ NPs 25 nm (−), SiO_2_ NPs 25 nm (+), and green SiO_2_ NPs for 24 h at 1 mg/mL and 5 mg/mL for 24 h and 48 h. After treatments, the cells were first lysed by the buffer provided in the assay kit to collect their intracellular contents. The enzyme activity was measured on cell lysates adding caspase-specific peptide that is conjugated to the p-nitroaniline (pNA). The caspase was cleaved by the peptide releasing the chromophore pNA. The latter was quantitated at 450 nm by a spectrophotometer. Data were expressed as mean ± SD.

### 2.11. Confocal Analysis

A549 cells were seeded in a 24-well plate at a concentration of 10^5^ cells/well and successively incubated with SiO_2_ NPs 110 nm (−), SiO_2_ NPs 110 nm (+), SiO_2_ NPs 50 nm (−), SiO_2_ NPs 50 nm (+), SiO_2_ NPs 25 nm (−), SiO_2_ NPs 25 nm (+), and green SiO_2_ NPs for 24 h at 1 mg/mL and 5 mg/mL for 24 h. After treatment, for each time point, the DMEM was removed, and the cells were washed with PBS and successively fixed with 0.25% glutaraldehyde (v/v) for 20 min. Finally, cells were permeabilized with 0.1% Triton X (v/v) for 10 min. The actin fibers were stained with FITC-phalloidin at a concentration of 1 *μ*g/mL overnight. Nuclei were labeled by DAPI at a concentration of 1 *μ*g/mL for 10 min. Laser scanning confocal microscopy was used on a Zeiss LSM700 (Zeiss) confocal microscope equipped with an Axio Observer Z1 (Zeiss) inverted microscope using ×100, 1.46 numerical aperture oil immersion lens for imaging. Confocal data were processed using ZEN2010 software (Zeiss).

The article "High Doses of Silica Nanoparticles Obtained by Microemulsion and Green Routes Compromise Human Alveolar Cells Morphology and Stiffness Differently" was published in 2022. Journal: Bioinorg Chem Appl.

### 2.12. Morphometric Quantification Parameters on Actin and Nuclei of A549 Cells

The morphometric quantifications (actin coherency, nuclear density, and nuclear morphology) were performed on confocal acquisitions using the ImageJ 1.47 software. The coherency parameter was calculated using the OrientationJ plugin manually selecting the cytoskeletal areas [32]. Nuclear morphology and density were quantified by means of Shape Descriptor and Integral Density tools [33]. The values of morphometric parameters were expressed as mean values, and their relative standard deviation was calculated on 30 different cells for each treatment.

### 2.13. Atomic Force Microscopy (AFM) Analysis

#### 2.13.1. Preparation of Samples

A549 cells were seeded in plastic Petri dishes at a concentration of 10^3^ cells/well. After 24 h, SiO_2_ NPs (5 mg/mL) were added to the culture medium for 24 h. Afterward, the medium enriched with NPs was removed and gently washed three times using PBS. Then, L15 medium was added.

#### 2.13.2. AFM Experiments

Indentation force curves were gained in force-volume (FV) mode by using a Bioscope Catalyst Atomic Force Microscope (Bruker Inc., CA, USA) implemented on an inverted optical microscope (Zeiss Observer Z1, Zeiss, Germany). All experiments were performed using Silicon Nitride V-shaped Bruker's Sharp Microlever (MSNL, tip C, Bruker Inc., CA, USA), having a nominal spring constant of 0.01 N/m. Prior to performing each measurement, the cantilever spring constant was determined with high precision, according to the thermal tune method [34]. The FV mapping was acquired 50 *μm∗*50 *μ*m areas, setting the acquisition parameters as ramp rate 4.88 Hz, FV scan rate 0.03 Hz, and Trigger Threshold 50 nm. The resolution of the FV topography acquisition channel was fixed at 64 (sample per line) × 64 (lines) to reduce the acquisition time and avoid deterioration of the living sample but it is still able to visualize the cell bodies. This condition was fundamental because 10 force-indentation curves were manually selected on 20 different cells for each treatment. These curves were analyzed by Nanoscope Analysis software (Bruker Inc., CA, USA) to extract Young's modulus values, using the procedure described in previous works [35, 36].

The article "High Doses of Silica Nanoparticles Obtained by Microemulsion and Green Routes Compromise Human Alveolar Cells Morphology and Stiffness Differently" was published in 2022. Journal: Bioinorg Chem Appl.

## 3. Results and Discussion

SiO_2_ NPs are widely used in different kinds of applications; in particular, they are employed in nanomedicine for the easiness functionalization procedure using chemical groups [37] or other NPs [38, 39] and capability to host certain types of drugs in their *core* [40]. In general, SiO_2_ NPs were considered biocompatible due to their amorphous nature, which makes them very different from the SiO_2_ crystalline form. For their potential use as therapeutic agents, high doses are needed, especially in living organisms of a specific weight and tonnage [13]; however, prior to application, the assessment of their impact on cells is essential. With this in mind, we studied the alterations in an alveolar cell model, that is, A549, after SiO_2_ NPs exposure since the inhalation is one of the most important routes of entry in living organisms.

To develop a full study, we first synthetized three different sizes of SiO_2_ NPs by the microemulsion method, which permitted us to obtain monodispersed and stable NPs. The microemulsion route is a system of water, oil, and an amphiphile thermodynamically stable [41]. We used quaternary and ternary microemulsion to obtain SiO_2_ NPs having larger sizes (110 nm and 50 nm) and 25 nm, respectively.

TEM images (Figures 4(a)–4(c)) confirmed the diameters of SiO_2_ NPs. In particular, the NPs appeared to be perfectly spherical and monodispersed with amorphous nature, as shown by diffraction figures (Figures 4(d)–4(f)). The mean size distributions calculated using ImageJ software on 70 nanoobjects showed sizes of 110 ± 2 nm (Figure 4(g)), 49 ± 3 nm (Figure 4(h)), and 25 ± 2 nm (Figure 4(i)). Gaussian fitting for each type of NPs was performed.

The same analysis was conducted on SiO_2_ NPs obtained by the green route. Green synthesis is an alternative approach to the conventional chemical and physical syntheses of nanomaterials [42]. In the last years, a lot of inorganics nanomaterials have been obtained using plants and microorganisms as a source of reducing and capping agents [43–46]. However, many works showed no spherical materials [47, 48], with visible impurity due to the high organic content of biological extracts [49].

We used *Laurus nobilis*, a native plant from the Mediterranean area, containing several clusters of phytochemicals [50]. These molecules are directly involved as reducing agents for the eco-friendly synthesis of SiO_2_ NPs [51], making the process cheap, time-saving, and sustainable [52]. This is in contrast with the microemulsion approach, characterized by expensive processes and numerous washing steps carried out to remove the toxic surfactants, as well as carcinogen solvents present in the synthetic mix [53]. In addition, the quality of SiO_2_ NPs obtained was very similar to those synthetized by the microemulsion approaches. The use of *Laurus nobilis* is particularly interesting due to its well-known antioxidant properties determined by a high concentration of polyphenols (c.a. 22 mg/L) [54] compared to the other plants [55].

The article "High Doses of Silica Nanoparticles Obtained by Microemulsion and Green Routes Compromise Human Alveolar Cells Morphology and Stiffness Differently" was published in 2022. Journal: Bioinorg Chem Appl.

The TEM images (Figures 5(a) and 5(b)) reported the SiO_2_ NPs obtained by green approach; they presented ultrasmall size and spherical morphology; in addition, no reaction residuals were visualized around NPs, and their structure was amorphous (Figure 5(c)). The SiO_2_ NPs size distribution performed by ImageJ software measured a mean size of about (3.4 ± 2) nm (Figure 5(d)).

After this careful characterization, we used a fraction of each SiO_2_ NP obtained by microemulsion approach to attach the amino groups on their surface by APTES.

DLS measurements showed a SiO_2_ NPs size increase than those observed by TEM analysis (Table 1). This was probably due to the formation of some NPs aggregates in water, typical for the metal oxide NPs. Regarding the zeta potential analysis, the measurements confirmed the negative charge on the bare NPs of the three sizes, whereas the NPs functionalized by APTES exhibited a positive surface charge as expected.

The size of green SiO_2_ NPs obtained by DLS analysis was 4 ± 2 nm, confirming the TEM analysis. An increase in size, due to the adsorption of the serum proteins on the NPs surface, was measured when NPs were dissolved in DMEM, showing a size of 6 ± 4 nm (Table 2). This adsorption can be demonstrated also by the surface charge measurements: as assumed, the charge became more negative after DMEM addition.

The long-term stability of SiO_2_ NPs, assessed by DLS, showed that the size of NPs did not change up to the 6th day. After this time, some aggregation phenomena were observed due to the presence of serum, salts, and vitamins in the cell culture medium (Figure 6).

Following the characterization of the SiO_2_ NPs in terms of physicochemical properties, we investigated their potential cytotoxic effect on the A549 cell line and the subsequential alterations on cellular compartments; these types of cells are the best model to simulate the impact of NPs on airways. For this purpose, we incubated the A549 cells with two concentrations of SiO_2_ NPs, 1 mg/mL, and 5 mg/mL, for 24 h and 48 h.

After 24 h, the lower concentration did not induce notable variations in terms of viability; however, higher toxicity was observed in the cells exposed to SiO_2_ NPs 25 (−). This effect became particularly evident using SiO_2_ NPs 25 (+); the trend was already visible after 24 h (Figure 7(a)) and 48 h (Figure 7(b)) of exposure.

The article "High Doses of Silica Nanoparticles Obtained by Microemulsion and Green Routes Compromise Human Alveolar Cells Morphology and Stiffness Differently" was published in 2022. Journal: Bioinorg Chem Appl.

In addition, the adverse effects observed were also dependent on the dosage applied. Using the highest concentration of SiO_2_ NPs 25 (−) and SiO_2_ NPs 25 (+), a strong reduction in the cell viability after 48 h was observed. In fact, using 1 mg/mL, the percentage of living cells was 42%; this value became 35% using 5 mg/mL. The 110 (−), 110 (+), 50 (−), and 50 (+) SiO_2_ NPs induced lower toxicity, but, as reported in the data above, the positively charged NPs were more able to trigger adverse effects in cells.

The SiO_2_ NPs achieved by the green route appeared to be more tolerated by A549 cells (Figure 7(c)) compared to NPs obtained by microemulsion using the same concentrations in time and dose-dependent manner.

After 48 h of exposure to green SiO_2_ NPs (5 mg/mL), most cells remained vital (about 70%). This trend was similar to the one observed for 110 and 50 nm NPs, in contrast with the idea that the smaller NPs are more harmful. This could be attributed to the green route that permitted us to obtain high-quality SiO_2_ NPs suitable for medicine applications.

In order to understand if cell death was triggered by apoptosis, the caspase-3 production was evaluated as percentage released in cells compared to untreated cells. The activation of caspase-3, known as executioner caspase [56], caused serious effects on nuclei and DNA as well as on cytoskeleton and on the mechanical behavior of cells due to the activation of specific biochemical pathways [57–59]. With the exposure of A549 cells to 1 mg/mL and 5 mg/mL of SiO_2_ NPs 110 nm (−), SiO_2_ NPs 110 nm (+), SiO_2_ NPs 50 nm (−), SiO_2_ NPs 50 nm (+), SiO_2_ NPs 25 nm (−), SiO_2_ NPs 25 nm (+), and green SiO_2_ NPs for 24 h and 48 h (Figure 7(d)), we observed caspase-3 stimulation enhancement compared with the control cells (8% ± 3).

The obtained results were in close agreement with the viability assays reported above. Sure enough, the caspase-3 stimulation was more pronounced using small-size SiO_2_ NPs in a dose- and time-dependent mode. Also in this case, the positive charged SiO_2_ NPs were more critical in terms of adverse effects induction. In particular, the SiO_2_ NPs 50 nm (+), SiO_2_ NPs 25 nm (−), and SiO_2_ NPs 25 nm (+) showed a value of 138% ± 6, 141% ± 8, and 145% ± 3, respectively, after 48 h using 5 mg/mL. Surprisingly, the SiO_2_ NPs obtained by the green approach exhibited values like the SiO_2_ NPs 50 nm (−), that is, about 125%. These results deviated from the notion that smaller NP_S_ are more toxic adding other pieces of knowledge in using ultrasmall NPs in the clinical application without dangerous effects. Contrary to the large NPs, the ultrasmall SiO_2_ NPs have great ability to improve plasmatic half-life, intensifying hepatobiliary clearance [60, 61]; therefore, they are suitable for real-time image-guided detection, localization, and surgical treatment of tumor cells [62, 63].

The article "High Doses of Silica Nanoparticles Obtained by Microemulsion and Green Routes Compromise Human Alveolar Cells Morphology and Stiffness Differently" was published in 2022. Journal: Bioinorg Chem Appl.

The cell death and apoptosis activation were correlated with the uptake capability. We analyzed the potential different internalization in A549 following the uptake of SiO_2_ NPs 110 (−), SiO_2_ NPs 110 (+) SiO_2_ NPs 50 (−) SiO_2_ NPs 50 (+), SiO_2_ NPs 25 (−), SiO_2_ NPs 25 (+), and green SiO_2_ NPs using the higher concentration tested in the previous experiments, namely, 5 mg/mL for 24 h and 48 h (Figure 8). After 24 h, the values of Si ranged from about 6 to 7 *μ*g when cells were treated with SiO_2_ NPs 110 nm (−), SiO_2_ NPs 110 nm (+), SiO_2_ NPs 50 nm (−) SiO_2_ NPs 50 nm (+), and SiO_2_ NPs 25 nm (−). The SiO_2_ NPs 25 (+) and green SiO_2_ NPs appeared to be more accumulated (Figure 8(a)). The Si content recorded after 48 h (Figure 8(b)) showed that the accumulation increased when size decreased, and it was greater using SiO_2_ NPs (+) and green NPs. Then, the low toxicity of green NPs did not depend on their higher accumulation compared to the others obtained by the microemulsion route.

The caspase-3 stimulation induces adverse effects on chromatin condensation, triggering a “cap-shaped” chromatin margination that is one of the first pieces of evidence of cellular apoptosis [64, 65]. In addition, the nuclei undergo fragmentation phenomena inducing micronuclei formation, which are often released into the cytosol or extracellular microenvironment, damaging also cellular membrane [66].

To fully understand this process, confocal analysis was performed to correlate the caspase-3 activation to the alterations in nuclear morphology after NPs exposure at a concentration of 5 mg/mL (Figure 9).

In detail, the SiO_2_ NPs (−) and SiO_2_ NPs (+) did not provoke significant changes in nuclear morphology (Figures 9(b) and 9(c)) compared to the control (Figure 9(a)), although the positive charged NPs exhibited slight alterations. The A549 cells incubated with SiO_2_ NPs 50 (−), SiO_2_ NPs 50(+), SiO_2_ NPs 25(−), and SiO_2_ NPs 25 (+) showed several morphological damage, including the presence of micronuclei (Figures 9(d)–9(g)). These effects were more pronounced when smaller and positive NPs were employed. Green SiO_2_ NPs induced mild nuclei modifications without micronuclei production, which were similar to those exposed to SiO_2_ NPs 110 nm (+) (Figure 9(h)).

Confocal acquisitions were analyzed by ImageJ software in order to quantify nuclear morphometric parameters, which could be critical to establishing cell health [33]; in detail, circularity, roundness, and nuclear area, as well as the nucleus/cytoplasm (N/C) ratio and fluorescence integrated density, were estimated (Figure 10).

The article "High Doses of Silica Nanoparticles Obtained by Microemulsion and Green Routes Compromise Human Alveolar Cells Morphology and Stiffness Differently" was published in 2022. Journal: Bioinorg Chem Appl.

Circularity and roundness are similar shape descriptor parameters that compare an object to a circle. In detail, roundness is the ratio between major and minor axes of an object; its value ranges from 0 to 1, corresponding to an infinitely elongated and perfectly circular object, respectively. Circularity indicates the degree of similarity to a perfect circle, ranging from 0 to 1 (for a perfect circle); this parameter is sensitive to the presence of irregularities on the object contour [67]. The typical circular nuclear morphology of untreated A549 cells was preserved following exposure to SiO_2_ NPs 110 (−) and SiO_2_ NPs 110 (+), as well as to SiO_2_ NPs 50 (−); on the other hand, the roundness exhibited a significant reduction in A549 exposed to SiO_2_ NPs 110 (+), due to the irregularities formed on the nuclei contours. The roundness reduction became more pronounced when the size of SiO_2_ NPs decreased or, in the case of the same size, in the presence of a positive charge (Figure 10(a)). In addition, after exposure to SiO_2_ NPs, nuclei area became smaller, and the effect was more evident when cells were incubated with SiO_2_ NPs 25 nm (+) and green SiO_2_ NPs showing values of about 98 *μ*m^2^ and 70 *μ*m^2^ respectively (Figure 10(b)). On the contrary, the percentage of nuclear/cytoplasm ratio became larger (Figure 10(c)); this meant that the cells underwent a shrinkage after treatment while their nuclei became proportionally larger. The impact on the reorganization of chromatin within the nucleus was higher when the size of the SiO_2_ NPs decreased and the surface charge was positive. The exposure to the green SiO_2_ NPs did not affect the N/C ratio in a significant manner (Figure 10(c)).

The obtained results were linked to the fluorescence nuclear density measurements that referred to the amount of chromatin in terms of fluorescence. This parameter was evaluated as integrated density (expressed as a percentage compared to the control, indicated as 100%), revealing a reduction of more than 20% for NPs with a size smaller than 110 nm (+) (Figure 10(d)).

The spatial reorganization of the nuclear body is strictly correlated with cytoskeleton reorganization [68], in particular through the actin fibers. Then, we analyzed the actin fiber conformation on the A549 cell lines (Figure 11), showing several differences between untreated (Figure 11(a)) and cells treated with NPs at 5 mg/mL. In detail, the treatment with SiO_2_ NPs 110 (−) (Figure 11(b)) and SiO_2_ NPs 110 (+) (Figure 11(c)) did not trigger evident alterations on actin fibers that were very similar to the control displaying a pebble-like shape, aligned actin fibers, and cell-cell adhesion [69]. In addition, in control cells, F-actin filaments were distributed on the whole apical surface. Instead, when the cells were treated with a smaller size of SiO_2_ NPs, a conformational cytoskeleton alteration was observed; the actin fibers were mostly localized on the edges of the cellular body. These remodulations were more recognizable in cells treated with SiO_2_ NPs 50 nm (−) (Figure 11(d)), SiO_2_ NPs 50 nm (+) (Figure 11(e)), SiO_2_ NPs 25 nm (−) (Figure 11(f)), and SiO_2_ NPs 25 nm (+) (Figure 11(g)); also in this case, the positive charge induced more adverse effects decreasing the cell-cell contacts. The treatment with green SiO_2_ NPs did not alter cell morphology in several manners (Figure 11(h)): this result was in line with the data previously obtained regarding the stimulation of caspase-3 production.

The article "High Doses of Silica Nanoparticles Obtained by Microemulsion and Green Routes Compromise Human Alveolar Cells Morphology and Stiffness Differently" was published in 2022. Journal: Bioinorg Chem Appl.

The altered organization of the actin network after NPs exposure was quantified by coherency parameter using ImageJ software (Figure 12). Its value is defined by the structure tensor, which quantifies the local orientation in a selected area of a specific image [33]; coherency values range from 0 to 1, corresponding to total isotropic orientation and highly oriented structures, respectively.

In confocal acquisition, F-actin fibers of untreated cells appeared to be locally ordered; however, they did not possess a privileged direction of orientation over the entire cell body, as confirmed by coherency estimation, which was about 0.43. The SiO_2_ NPs 110 (+) and 110 (−) treatments induced a slight modification of the actin network, corresponding to a coherency roughly equal to 0.38 and 0.36, respectively. Cells exposed to the smaller size (SiO_2_ NPs 50 nm and 25 nm) clearly showed the loss of fibers organization. The positive surface reduced the coherency in a strong manner, reporting values of about 0.18 and 0.1 for SiO_2_ NPs 50 (+) nm and SiO_2_ NPs 25 (+) nm; the data were perfectly consistent with the confocal images.

Finally, in the case of green NPs, we observed an organization of actin comparable to values associated with the SiO_2_ NPs (−). As a matter of fact, cortical network defragmentation, local circular thickening, and protrusions were visible but still ensured cell-cell contact.

Hence, the cytoskeleton plays several essential functions modulating the cellular architecture. In addition, it senses/transmits mechanical stimuli from/to neighboring cells and microenvironment, regulating in turn (i) the cellular overall shape and the spatial organization of the subcellular organelles, (ii) cellular dynamics, and (iii) motility [70, 71]. Any alteration of the cytoskeleton induces and/or corresponds to cell damage [72]. In particular, the damaged cytoskeletal organization is linked to an altered mechanical behavior that is involved in numerous cellular pathways, such as migration, differentiation, wound healing, and cancer metastasis [73]. Following these observations, the cellular mechanical properties represent a key factor to define the cellular health condition.

The article "High Doses of Silica Nanoparticles Obtained by Microemulsion and Green Routes Compromise Human Alveolar Cells Morphology and Stiffness Differently" was published in 2022. Journal: Bioinorg Chem Appl.

The experiments presented investigate the biophysical property alterations in cells exposed to SiO_2_ NPs.

With this in mind, we believe that the evaluation of potential cytotoxicity of NPs should strongly consider the biomechanical assessment to integrate information obtained by conventional viability assays. In general, the cell membrane elasticity is expressed in terms of Young's modulus [74, 75]. When this parameter is altered due to actin rearrangements, some diseases can arise; for this reason, elasticity can be defined as an indicator of possible pathological states [25].

Then, we carefully measured Young's modulus of the A549 cellular membrane, following the exposure to the different types of SiO_2_ NPs using a concentration of 5 mg/mL for 24 h. The data were obtained through indentation experiments conducted by AFM in force-volume mode and living conditions. The AFM analysis permitted us to acquire topography (Figure 13) and, at the same time, the force-distance curves in correspondence of each pixel for control cells (Figure 13(a)), SiO_2_ NPs 110 nm (−) (Figure 13(b)), SiO_2_ NPs 110 nm (+) (Figure 13(c)), SiO_2_ NPs 50 nm (−) (Figure 13(d)), SiO_2_ NPs 50 nm (+) (Figure 13(e)), SiO_2_ NPs 25 nm (−) (Figure 13(f)), SiO_2_ NPs 25 nm (+) (Figure 13(g)), and green SiO_2_ NPs (Figure 13(h)).

Cellular Young's modulus values obtained by analysis of the collected curves are reported in Figure 14. We observed several changes in terms of elasticity after NPs incubation, especially for small and positive charged NPs. In detail, the evaluation of Young's moduli in control A549 cells showed a value of (8.55 ± 0.05) kPa (Figure 14(a)) that decreased after SiO_2_ NPs exposure becoming equal to 8.22 ± 0.07 kPa, 7.6 ± 0.1 kPa, and 5.1 ± 0.1 kPa, in A549 treated with 110 nm (−), 50 nm (−), and 25 nm (−) SiO_2_ NPs, respectively (Figures 14(b), 14(d), and 14(f)). When cells were exposed to the positive charged SiO_2_ NPs, Young's modulus reduction became more pronounced: the elasticity values were 8.11 ± 0.09 kPa, 6.1 ± 0.1 kPa, and 3.6 ± 0.05 kPa after SiO_2_ NPs 110 nm (+), 50 nm (+), and 25 nm (+) exposure (Figures 14(c), 14(e), and 14(g)). This result suggested the role of SiO_2_ NPs exposure on A549 force-deformation profiles deeply dependent on the NPs size. Additionally, the NPs surface functionalization enhanced their cytotoxic potential, confirming the results obtained by biological assays. Finally, Young's modulus value equal to 6.00 ± 0.1 kPa was obtained in A549 cells exposed to green SiO_2_ NPs (Figure 14(h)); this datum demonstrated that the green route permitted us to obtain very small NPs (about 4 nm) with effects similar to the same nanoobjects having bigger size also in terms of elasticity.

The article "High Doses of Silica Nanoparticles Obtained by Microemulsion and Green Routes Compromise Human Alveolar Cells Morphology and Stiffness Differently" was published in 2022. Journal: Bioinorg Chem Appl.

In general, we asserted that the decrease of Young's modulus values stimulated by NPs exposure was associated with the elasticity enhancement; cells became softer with respect to the untreated cells. The softer cell profile can impact the physiological homeostasis of cells perturbing some cellular pathways associated with the actin remodulation and coherency decrease. In particular, the increase of elasticity is involved in cancer progression due to the cell junctions destroying and the consequent metastatization [17, 76]. Therefore, according to this evidence, the green SiO_2_ NPs did not induce significant variations in terms of elasticity, thus making them useable even at high doses in living systems.

## 4. Conclusion

In this experimental work, we tested high doses of monodispersed SiO_2_ NPs with different size on A549 cells, being the best model to simulate an inhalation route. Certainly, their massive use in various fields requires the evaluation of their toxicity at high concentrations. We obtained bare SiO_2_ NPs with a negative charge (110 nm, 50 nm, and 25 nm) using the microemulsion approach and the correspondent sizes positive charged. We also developed a one-pot eco-friendly route to obtain monodisperse SiO_2_ NPs having small size using leaves extract.

We tested their toxicity in A549 cells through biological assays using 1 mg/mL and 5 mg/mL of concentrations. The data suggested that the smallest and positive charged NPs, achieved from the microemulsion approach, were more toxic for cells than the larger ones. Surprisingly, the green SiO_2_ NPs did not induce intense toxicity, despite the fact they were ultrasmall (c.a. 4 nm) and highly internalized. The modifications on nuclei and actin fibers morphology were evaluated, showing that the rearrangement of the cytoskeleton due to the NPs exposure was closely connected with the nuclei. These cellular comparts were correlated with the activation of apoptosis through the caspase-3 stimulation.

The article "High Doses of Silica Nanoparticles Obtained by Microemulsion and Green Routes Compromise Human Alveolar Cells Morphology and Stiffness Differently" was published in 2022. Journal: Bioinorg Chem Appl.

Finally, we investigated the cytotoxic potential of different SiO_2_ NPs from a mechanical point of view using AFM. Following the NPs uptake, the membrane elasticity change was assessed. This analysis demonstrated that the smaller SiO_2_ NPs derived from microemulsion synthesis increased the membrane elasticity. The cells exposed to green SiO_2_ NPs, despite their smaller size (c.a. 4 nm), exhibited elasticity values comparable to larger NPs, confirming data obtained in biological assays. Then, the use of high doses of green SiO_2_ NPs did not trigger relevant effects in cells, also removing the possibility that these materials could induce malignant transformation in cells, often associated with the soft cell membrane. For this reason, these new nanostructures are promising materials able to induce low toxicity compared to the larger ones. In addition, their ultrasmall size can promote a high internalization rate, which is important to deliver high doses of drugs in specific sites. Our next experiments will be focused on green SiO_2_ NPs functionalization modulation in order to develop safe nanotools specific to a different biological target.

## Figures and Tables

**Figure 1:** Schematic representation of SiO_2_ NPs obtained by the microemulsion method.

**Figure 2:** Schematic representation of SiO_2_ NPs functionalization with APTES.

**Figure 3:** Schematic representation of SiO_2_ NPs green synthesis.

**Figure 4:** Representative TEM images of SiO_2_ NPs 110 nm (a), SiO_2_ NPs 50 nm (b), and SiO_2_ NPs 25 nm (c), and related diffraction figures (d–f). Statistical analysis with Gaussian fit (blue line) SiO_2_ NPs 110 nm (g), SiO_2_ NPs 50 nm (h), and SiO_2_ NPs 25 nm (i). The scale bar of (a), (b), and (c) is 200 nm.

**Figure 5:** Representative TEM images of green SiO_2_ NPs at two different magnifications, (a) scale bar 100 nm and (b) scale bar 50 nm, and the related diffraction figures (c). Statistical analysis with Gaussian fit (blue line) (d).

**Figure 6:** Stability studies of SiO_2_ NPs 110 (−), SiO_2_ NPs 110 (+), SiO_2_ NPs 50 (−), SiO_2_ NPs 50 (+), SiO_2_ NPs 25 (−), and SiO_2_ NPs 25 (+) in DMEM acquired after 0, 3, 6, 9, and 12 days. The measurements were performed using the DLS technique.

**Figure 7:** Viability assay (WST-8) of A549 cell lines after 24 h (a) and 48 h (b) of exposure to 1 mg/mL and 5 mg/mL of SiO_2_ NPs 110 nm (−), SiO_2_ NPs 110 nm (+), SiO_2_ NPs 50 nm (−), SiO_2_ NPs 50 nm (+), SiO_2_ NPs 25 nm (−), and SiO_2_ NPs 25 nm (+). Viability assay (WST-8) of A549 cell lines after 24 h and 48 h of exposure to 1 mg/mL and 5 mg/mL of green SiO_2_ NPs (c). The viability of NP-treated cells was normalized to nontreated control cells. As a positive control (P), the cells were exposed to 5% DMSO (data not shown). Data reported as the mean ± SD from three independent experiments are considered statistically significant, compared with the control (*n* = 8) for *p* value < 0.05 (<0.05^*∗*^). Effect of SiO_2_ NPs 110 nm (−), SiO_2_ NPs 110 nm (+), SiO_2_ NPs 50 nm (−), SiO_2_ NPs 50 nm (+), SiO_2_ NPs 25 nm (−), SiO_2_ NPs 25 nm (+), and green SiO_2_ NPs on levels of apoptosis (d). Caspase-3 assay was performed incubating A549 cells with 1 mg/mL and 5 mg/mL of NPs for 24 h and 48 (h). Data are reported as mean ± SD from three independent experiments; ^*∗*^*p* < 0.05 compared with control (*n* = 3).

The article "High Doses of Silica Nanoparticles Obtained by Microemulsion and Green Routes Compromise Human Alveolar Cells Morphology and Stiffness Differently" was published in 2022. Journal: Bioinorg Chem Appl.

**Figure 8:** Elemental analysis performed in A549 cell lines exposed to 5 mg/mL of SiO_2_ NPs 110 nm (−), SiO_2_ NPs 110 nm (+), SiO_2_ NPs 50 nm (−), SiO_2_ NPs 50 nm (+), SiO_2_ NPs 25 nm (−), SiO_2_ NPs 25 nm (+), and green SiO_2_ NPs. Cells were then harvested and counted, and Si content was measured in 360.000 cells (*μ*g Si). Histograms reported the silicon amount. Data were reported as mean ± SD from three independent experiments: statistical significance of exposed cells versus control cells (0 ug) for *p* value < 0.05 (<0.05^*∗*^).

**Figure 9:** Representative confocal images of untreated A549 cells (a) and cells exposed to 5 mg/mL of SiO_2_ NPs 110 nm (−) (b), SiO_2_ NPs 110 nm (+) (c), SiO_2_ NPs 50 nm (−) (d), SiO_2_ NPs 50 nm (+) (e), SiO_2_ NPs 25 nm (−) (f), SiO_2_ NPs 25 nm (+) (g), and green SiO_2_ NPs (h) on A549 nuclei after 48 h. The cells were fixed and then stained with DAPI. Images were acquired using a Zeiss LSM700 (Zeiss) confocal microscope, equipped with an Axio Observer Z1 (Zeiss) inverted microscope, using a ×100, 1.46 numerical aperture oil immersion lens. All data were processed using the ZEN software.

**Figure 10:** Histograms reported the mean values and their respective standard deviation of shape parameter index (circularity and roundness) (a), nuclear area (b), nucleus/cytoplasm ratio (N/C) (c), and nuclear fluorescence density (d). The statistical significance of results compared to the control cells was evaluated by Student's *t*-test and reported in histograms for ^*∗∗*^*p* < 0.001.

**Figure 11:** Representative confocal images of untreated A549 cells (a) and cells exposed to 5 mg/mL of SiO_2_ NPs 110 nm (−) (b), SiO_2_ NPs 110 nm (+) (c), SiO_2_ NPs 50 nm (−) (d), SiO_2_ NPs 50 nm (+) (e), SiO_2_ NPs 25 nm (−) (f), SiO_2_ NPs 25 nm (+) (g), and green SiO_2_ NPs (h) on A549 nuclei for 24 h. Then, cells were fixed and then stained with FITC-phalloidin for actin and DAPI for nuclei. 2D images of cortical actin were acquired using a Zeiss LSM700 (Zeiss) confocal microscope.

The article "High Doses of Silica Nanoparticles Obtained by Microemulsion and Green Routes Compromise Human Alveolar Cells Morphology and Stiffness Differently" was published in 2022. Journal: Bioinorg Chem Appl.

**Figure 12:** Coherency values calculated on A549 confocal acquisitions. Data were expressed as the mean value and relative SD using ImageJ (calculation on 15 cells). The mean values and their standard deviations are reported in the histograms. Data were statistically significant for ^*∗∗*^*p* < 0.001.

**Figure 13:** Representative AFM height channel acquisitions performed in force-volume mode on living A549 cells (a) and cells exposed to 5 mg/mL of SiO_2_ NPs 110 nm (−) (b), SiO_2_ NPs 110 nm (+) (c), SiO_2_ NPs 50 nm (−) (d), SiO_2_ NPs 50 nm (+) (e), SiO_2_ NPs 25 nm (−) (f), SiO_2_ NPs 25 nm (+) (g), and green SiO_2_ NPs (h) for 24 h.

**Figure 14:** Young's modulus distributions with Gaussian fit functions (blue line). Control A549 cells (a) and cells exposed to 5 mg/mL of SiO_2_ NPs 110 nm (−) (b), SiO_2_ NPs 110 nm (+) (c), SiO_2_ NPs 50 nm (−) (d), SiO_2_ NPs 50 nm (+) (e), SiO_2_ NPs 25 nm (−) (f), SiO_2_ NPs 25 nm (+) (g), and green SiO_2_ NPs (h) for 24 h.

**Table 1:** Characterization of SiO_2_ NPs 110 (−), SiO_2_ NPs 110 (+) SiO_2_ NPs 50 (−), SiO_2_ NPs 50 (+), SiO_2_ NPs 25 (−), and SiO_2_ NPs 25 (+) in water and DMEM by DLS and *ζ*-potential measurements.

Samples in water	Size (nm) ± SD	*ζ*-Potential (mV) ± SD
SiO_2_ NPs 110 (−)	120 ± 5	−8 ± 2
SiO_2_ NPs 110 (+)	125 ± 4	+12 ± 3
SiO_2_ NPs 50 (−)	55 ± 2	−16 ± 4
SiO_2_ NPs 50 (+)	65 ± 3	+16 ± 2
SiO_2_ NPs 25 (−)	28 ± 5	−15 ± 3
SiO_2_ NPs 25 (+)	33 ± 7	+11 ± 3
Samples in DMEM	Size (nm)	*ζ*-Potential (mV)
SiO_2_ NPs 110 (−)	128 ± 4	−15 ± 2
SiO_2_ NPs 110 (+)	132 ± 6	+20 ± 5
SiO_2_ NPs 50 (−)	62 ± 4	−24 ± 4
SiO_2_ NPs 50 (+)	63 ± 6	+30 ± 2
SiO_2_ NPs 25 (−)	37 ± 5	−21 ± 6
SiO_2_ NPs 25 (+)	35 ± 7	+33 ± 5

**Table 2:** Characterization in water and DMEM of SiO_2_ NPs 110 (−), SiO_2_ NPs 110 (+), SiO_2_ NPs 50 (−), SiO_2_ NPs 50 (+), SiO_2_ NPs 25 (−), and SiO_2_ NPs 25 (+) by DLS and *ζ*-potential measurements.

Sample in water	Size (nm) ± SD	*ζ*-Potential (mV) ± SD
Green SiO_2_ NPs	4 ± 1	−12 ± 5
Sample in DMEM	Size (nm)	*ζ*-Potential (mV)
Green SiO_2_ NPs	6 ± 4	−22 ± 3

## Data Availability

The data presented in this study are included in this article.
